# The Design of Individual Orthopedic Insoles for the Patients with Diabetic Foot Using Integral Curves to Describe the Plantar Over-Pressure Areas

**DOI:** 10.1155/2021/9061241

**Published:** 2021-08-06

**Authors:** Merab Shalamberidze, Zaza Sokhadze, Malvina Tatvidze

**Affiliations:** ^1^Department of Design and Technology, Akaki Tsereteli State University, 59, Tamar Mepe Str., Kutaisi, Georgia 4600; ^2^Department of Mathematics, Akaki Tsereteli State University, 59, Tamar Str., Kutaisi, Georgia 4600; ^3^Department of Chemical and Environmental Technologies, Akaki Tsereteli State University, 59, Tamar Mepe Str., Kutaisi, Georgia 4600

## Abstract

Identification of over-pressure areas in the plantar side of the foot in patients with diabetic foot and reduction of plantar pressure play a major role in clinical practice. The use of individual orthopedic insoles is essential to reduce the over-pressure. The aim of the present study is to mark the over-pressure areas of the plantar part of the foot on a pedogram and describe them with high accuracy using a mathematical research method. The locally over-pressured areas with calluses formed due to repeated injuries were identified on the patients' pedograms. The geometric shapes of the over-pressure areas were described by means of the integral curves of the solutions to Dirichlet singular boundary differential equations. Based on the mathematical algorithm describing those curves, the computer programs were developed. The individual orthopedic insoles were produced on a computer numerical control milling machine considering the locally over-pressured areas. The ethylene vinyl acetate polymers of different degrees of hardness were used to produce the individual orthopedic insoles. For the over-pressure areas, a soft material with a hardness of 20 Shore A was used, which reduces the pressure on the plantar side of the foot and increases the contact area. A relatively hard material with a hardness of 40 Shore A was used as the main frame, which imparts the stability of shape to the insole and increases its wear life. The individual orthopedic insoles produced by means of such technology effectively reduce the pressure on the plantar side of the foot and protect the foot from mechanical damage, which is important for the treatment of the diabetic foot.

## 1. Introduction

Based on the biomechanics of human movement, the feet are the basis of the musculoskeletal system. During walking, the foot performs complex mechanical movements and its bone system and soft tissues are over-pressured. In particular, the plantar side, heel, and metatarsophalangeal (MTP) joints are over-pressured. The patients with diabetes mellitus develop skin maceration, bruises, calluses, and other pathological changes on the locally over-pressured areas, which remain undetected due to diminution/loss of pain, temperature, and tactile sensations. On the injured areas, an ulcer develops, which is easily infected [1].

Diabetic foot ulcer, gangrene, and amputation cause great harm to the patient's health, lower the quality of their life, and lead to premature disability. Patients often need repeated surgical intervention [2]. It should be noted that in Georgia, about 60% of patients with diabetic foot syndrome are aged 35 to 65 constituting the most productive part of the labor force, who can bring a great benefit to the country.

In patients with diabetes mellitus especially in patients with diabetic foot syndrome, it is necessary to use the orthopedic individual foot protectors for prophylaxis and treatment. There is no other alternative [3, 4].

The treatment of diabetic foot using the individual orthopedic insoles is a proven method in the developed world, which is reflected in the studies of many scientists.

Paper [5] considers the peak pressure, as the measure traditionally used in the studies evaluating the effect of offloading of the plantar over-pressure areas. In paper [6], prescription of medical-grade footwear including custom-made in-shoe orthoses or insoles for people with a foot deformity or preulcerative lesion is discussed. The study in [7] is focused on understanding the pressure relieving effects of orthotic insoles designed for inside retail footwear and targeted at people with diabetes and the risk of the first forefoot ulceration. The paper [8] considers the effects of diabetic therapeutic footwear on preventing the ulcer recurrence in patients with diabetic foot. Orthopedic insoles are developed to support the medial longitudinal and lateral arch and partly transfer the pressure away from the forefoot and heel, to relieve the pressure on the forefoot and heel. The effectiveness of different designs of orthopedic insoles and orthopedic shoe soles during the treatment of various forms of diabetic foot is discussed, and the relevance of measurements of plantar pressure in predicting ulceration for patients with diabetic foot is described in [9].

The description of complex geometric shapes using mathematical research methods is considered in the works of scientists. Objects with complex geometric shapes—foot and boot-tree—are of the greatest complexity for design [10, 11]. The description of the geometric shapes of the boot-tree is presented in the works [12, 13]. The paper [14] describes the construction of a shape of the orthopedic boot-tree print by means of the solution to a differential equation with deviating argument. The papers [15, 16] describe the construction of the orthopedic boot-tree using Dirichlet singular boundary differential equations.

Based on the analysis of the mathematical research methods, it was decided to describe the over-pressure areas of the plantar side of the foot by means of the integral curves of the solutions to Dirichlet singular boundary differential equations. Application of the mentioned method allows description of complex geometric forms with great accuracy. The other methods are characterized by some inaccuracies and are time consuming.

In the process of producing individual orthopedic insoles, considerable attention is paid to the selection of the materials for the insoles. The effectiveness of the use of different polymeric materials for reduction of the peak pressure on the plantar side of the foot is considered in [17]. In particular, the microporous polyurethane of medium and low densities was investigated, and it was established that both materials can partially reduce the peak pressure. The medium- and low-density ethylene vinyl acetate (EVA) polymers were also investigated. The use of those polymers significantly reduces the peak pressure on the plantar side of the foot and increases the contact area, which shows the advantages of using EVA polymers.

It should be noted that the description of locally over-pressured areas of the plantar side of the foot using the mathematical research methods are not considered in any work of the scientists.

Local pressure on the plantar side of the foot in patients with diabetic foot is individual according to the geometric shapes of the over-pressure areas. The use of the improperly designed insoles made from the material of homogeneous hardness in the treatment of diabetic foot causes mechanical damage to the over-pressure areas of the diabetic foot. The injured areas of the foot are easily infected, and a diabetic ulcer develops, which later can become the cause of the diabetes-related lower leg amputations.

In order to implement the right strategy for the diabetic foot treatment process, it is necessary to describe the over-pressure areas of the plantar side of the foot with high precision using the mathematical research methods, develop software packages based on the mathematical algorithm, and produce individual orthopedic insoles from combined materials on the computer numerical control (CNC) milling machine.

Given the global nature of the problem, the goal of the present work is to effectively reduce pressure on locally over-pressured areas on the plantar side of the diabetic foot and protect the foot from mechanical damage. To achieve the mentioned goal, the following were necessary:

- To study the plantar pressure in patients with diabetic foot using the pedograph method
- To register the locally over-pressured areas on the pedograms, where the pressure exceeds 200 kPa using curves
- To describe complex geometric shapes of over-pressure areas using the mathematical research methods
- To develop the complete software packages based on the mathematical algorithm
- To select the materials for producing orthopedic insoles
- To produce individual orthopedic insoles from the combined materials on a CNC milling machine considering locally over-pressured areas

## 2. Research Methods and Materials

### 2.1. Mathematical Research Method

An important novelty of the research is that the geometric shapes of the locally over-pressured areas for the individual orthopedic insoles were described by the integral curves of the solutions to Dirichlet singular boundary differential equations [18]:

(1) $$\begin{array}{c} u^{\prime \prime }\left(t\right)+\frac{a}{t}u^{\prime }\left(t\right)-\frac{a}{t^{2}}u\left(t\right)=f\left(t,u\left(t\right),u^{\prime }\left(t\right)\right), \end{array}$$

(2) $$\begin{array}{c} u\left(t\right)=0,u\left(T\right)=0, \end{array}$$

where *a* ∈ (−∞; 1), *f* satisfies the local Carathéodory condition for a set [0, *T*] × *D* ,*D* = (0; +∞) × *R*.

Lemma 3.1 in [11] clearly shows the solution to problems (1)–(2), particularly,

(3) $$\begin{array}{c} u\left(t\right)=c_{1}t+c_{2}t^{-a}+t\int_{t}^{T}S^{-a-2}\left(\int_{S}^{T}\xi^{a+1}f\left(t,u\left(\xi \right),u^{\prime }\left(\xi \right)d\xi \right)d\xi \right), \end{array}$$

where *c*_1_ *c*_2_ ∈ *π* *t* ∈ [0, *T*].

The goal of the present paper is to clearly write the solution to different cases of a function *f*(*t*, *u*(*t*), *u*′(*t*)) given on the right side of equation (1) and also to construct the integral curves of these solutions using formula (3) for different values of *a*. This method will allow accurately describing the shapes of the over-pressure zones of the plantar part of the foot.

Consider the first particular case for problems (1)–(2):

(4) $$\begin{array}{c} u^{\prime \prime }+\frac{2}{t}u^{\prime }-\frac{2}{t^{2}}u=t, \end{array}$$

(5) $$\begin{array}{c} u\left(1\right)=0\;u^{\prime }\left(1\right)=c, \end{array}$$

viz., with provision for *f*(*t*, *u*(*t*), *u*′(*t*)) = *t*, *a* = −2, and  *t* ∈ [0, 1], the solution of problem (4)–(5) is as follows:

(6) $$\begin{array}{c} u\left(t\right)=\frac{t^{3}}{2}-\frac{1}{3}ct^{-2}-\left(1-\frac{1}{3}c\right)t+\frac{1}{2}. \end{array}$$

If *c* = 0, then

(7) $$\begin{array}{c} u\left(t\right)=\frac{t^{3}}{2}-t+\frac{1}{2}. \end{array}$$

Figure 1 illustrates the appropriate integral curve graphics for the obtained solutions.

Consider the same case for problems (1)–(2):

(8) $$\begin{array}{c} u^{\prime \prime }+\frac{a}{t}u^{\prime }-\frac{a}{t^{2}}u=t^{2}, \end{array}$$

(9) $$\begin{array}{c} u\left(1\right)=0\;u^{\prime }\left(1\right)=c, \end{array}$$

viz., with provision of *f*(*t*, *u*(*t*), *u*′(*t*)) = *t*, *a* = −2, and*t* ∈ [0, 1], the solution of problems (8)–(9) is as follows:

(10) $$\begin{array}{c} u\left(t\right)=\left(-\frac{1}{3}-\frac{1}{3}c\right)t+\frac{1}{3}c\frac{1}{t^{2}}+\frac{2}{3}t-\frac{t^{2}}{2}+\frac{t^{4}}{6}. \end{array}$$

If *c* = 0, then

(11) $$\begin{array}{c} u\left(t\right)=\frac{t^{4}}{6}-\frac{t^{2}}{2}+\frac{1}{3}t. \end{array}$$

Figure 2 shows the graphics of the appropriate integral curves for the solutions obtained.

Thus, by means of the integral curves of the solution to the singular Dirichlet boundary value problem, it is possible to describe the over-pressure areas on the patient's pedograms with great accuracy.

Using this method of mathematical research, the surface frame of the individual orthopedic boot-tree is designed in 3D format [19, 20].

### 2.2. Pedograph Research Method

Pedographic study of patients with diabetic foot was carried out using a pedograph Emed -25 at/D manufactured by the Novel company (Munich, Germany).

The pedograph method provides important information about the dynamic pressure on the plantar side of the foot. That method is used for determining and recording the following parameters: distribution of pressure on the foot plantar surface, peak pressure, pressure during the feet locomotion, arch index, time of contact of the foot with the pedograph surface, and pressure-time integral. All the important measurement parameters are calculated automatically. Information is reflected as an image of the foot with different color spectra.

In the present research, the pedograph method was used to determine the distribution of plantar pressure in the patients with diabetes mellitus and to mark the over-pressure areas.

### 2.3. Materials

It should be noted that the design and construction of individual orthopedic insoles for patients with diabetic foot from a homogeneous material alone did not yield the desired result. For local pressures on the plantar side of the foot, it is necessary to select soft materials. Therefore, for effective treatment, it is necessary to combine soft (for locally over-pressured areas) and relatively rigid (for the main frame of the insole) materials to produce the individual orthopedic insoles.

In the process of production of the individual orthopedic insoles for over-pressure areas of the diabetic foot, the soft material was selected according to the personal sensations of the patient. They were offered EVA polymers of various degrees of hardness, namely, from 15 Shore A to 30 Shore A. The patient chose EVA polymer of 20 Shore A-strength.

EVA polymer with a hardness of 20 Shore A was used to produce the individual orthopedic insoles for over-pressure areas and EVA polymer with a hardness of 40 Shore A for the main frame.

## 3. Research Results

The insoles for the patients with diabetic foot were produced individually based on the data obtained from the foot pedography. The study involved patients diagnosed with diabetes mellitus, type 2; diabetic angiopathy; diabetic sensorimotor peripheral neuropathy; and diabetic foot. All patients had the calluses on the plantar side of the foot, particularly in the heel and metatarsophalangeal (MTP) joints, without ulcers and infections. All patients were overweight, with an average weight from 120 kg to 130 kg.

Figure 3 shows the pedogram of the patient with diabetic foot, 63, weighing 126 kg, with a body mass index 39.77 (class 2 obesity) and duration of illness of 12 years. The analysis of the pedogram shows that the main pressure falls on the areas of the heel and MTP joints of the foot plantar surface.

The areas marked in red on the pedogram represent the locally over-pressured areas, where the calluses developed due to repetitive injuries. Those areas are at risk of ulceration.

The locally over-pressured areas were marked with curves, which showed the pressure of 200 kPa and over. The curves in Figure 1 also show the over-pressure areas on the plantar side of the foot.

The shapes of the above curves were described by the integral curves of the solutions to Dirichlet singular boundary differential equations.

Figure 4 shows the shape of the curve of a locally over-pressured area in the right foot's MTP area, which was taken from the pedogram.

The curve shown in Figure 4 was preliminarily divided into nine parts to describe its shape. Each numbered section was described using the integral curves of solutions to the differential equations given below. Nine parts of the integral curves identically corresponding to the geometric shapes of the curve on the over-pressure area of the plantar side of the MTP of the right foot were chosen, particularly the following:

1. AB curve corresponds to that part of the solution to equation

(12) $$\begin{array}{c} u\left(t\right)=\left(-\frac{1}{3}-\frac{1}{3}c\right)t+\frac{1}{3}c\frac{1}{t^{2}}+\frac{2}{3}t-\frac{t^{2}}{2}+\frac{t^{4}}{6}, \end{array}$$

for which *c* = 0 and corresponds to a set [1; 0] × [2.2; 2.5]

(2) BC curve corresponds to that part of the solution to equation

(13) $$\begin{array}{c} u\left(t\right)=\frac{t^{3}}{2}-\frac{1}{3}{ct}^{-2}-\left(1-\frac{1}{3}c\right)t+\frac{1}{2}, \end{array}$$

for which *c* = 0 and corresponds to a set [−1.6; 0.1] × [−2.5; −3.55]

(3) CD curve corresponds to that part of the solution to equation

(14) $$\begin{array}{c} u\left(t\right)=\left(-\frac{1}{3}-\frac{1}{3}c\right)t+\frac{1}{3}c\frac{1}{t^{2}}+\frac{2}{3}t-\frac{t^{2}}{2}+\frac{t^{4}}{6}, \end{array}$$

for which *c* = 1 and corresponds to a set [−0.6; 0.4] × [−0.4; 2.8]

(4) DE curve corresponds to that part of the solution to equation

(15) $$\begin{array}{c} u\left(t\right)=\frac{t^{3}}{2}-\frac{1}{3}{ct}^{-2}-\left(1-\frac{1}{3}c\right)t+\frac{1}{2}, \end{array}$$

for which *c* = 5 and corresponds to a set [−0.3; −0.5] × [−0.5; −5.2]

(5) EF curve corresponds that part of the solution to equation

(16) $$\begin{array}{c} u\left(t\right)=\frac{t^{3}}{2}-\frac{1}{3}{ct}^{-2}-\left(1-\frac{1}{3}c\right)t+\frac{1}{2}, \end{array}$$

for which *c* = 2 and corresponds to a set [−0.6; −2.5] × [1; −4.1]

(6) FH curve corresponds to that part of the solution to equation

(17) $$\begin{array}{c} u\left(t\right)=\left(-\frac{1}{3}-\frac{1}{3}c\right)t+\frac{1}{3}c\frac{1}{t^{2}}+\frac{2}{3}t-\frac{t^{2}}{2}+\frac{t^{4}}{6}, \end{array}$$

for which *c* = 3 and corresponds to a set [2; −1.8] × [2.5; 1.45]

(7) HN curve corresponds to that part of the solution to equation

(18) $$\begin{array}{c} u\left(t\right)=\frac{t^{3}}{2}-\frac{1}{3}{ct}^{-2}-\left(1-\frac{1}{3}c\right)t+\frac{1}{2}, \end{array}$$

for which *c* = 0 and corresponds to a set [1.2; 0.1] × [2; 2.5]

(8) NP curve corresponds to that part of the solution to equation

(19) $$\begin{array}{c} u\left(t\right)=\frac{t^{3}}{2}-\frac{1}{3}{ct}^{-2}-\left(1-\frac{1}{3}c\right)t+\frac{1}{2}, \end{array}$$

for which *c* = 0 and corresponds to a set [2.3; 9.8] × [2.9; 4.5]

(9) PA curve corresponds to that part of the solution to equation

(20) $$\begin{array}{c} u\left(t\right)=\frac{t^{3}}{2}-\frac{1}{3}{ct}^{-2}-\left(1-\frac{1}{3}c\right)t+\frac{1}{2}, \end{array}$$

for which *c* = 0 and corresponds to a set [−0.1; 1] × [−1.3; 0.85]

Based on the above-mentioned mathematical algorithm, the software was developed to describe the curve sections. Further, by rotating and transferring these sections, the entire geometric shape of the curves was assembled to represent the locally over-pressured areas on the MTP area of the right foot's plantar surface. The exact image is shown in Figure 4.

Figure 5 geometrically shows the curve of the locally over-pressured regions in the heel area of the right foot, taken from the pedogram.

The curve was preliminarily divided into seven parts to describe its shape. Each numbered section was described using the integral curves of the solutions to differential equations given below. Ten parts of the integral curves identically corresponding to the geometric shapes of the curve of over-pressure area in the right foot's heel, particularly the following:

1. AB curve corresponds to that part of the solution to equation

(21) $$\begin{array}{c} u\left(t\right)=\frac{t^{3}}{2}-\frac{1}{3}{ct}^{-2}-\left(1-\frac{1}{3}c\right)t+\frac{1}{2}, \end{array}$$

for which *c* = 0 and corresponds to a set [0.1; 0, 4] × [−0.02; 0.1]

(2) BC curve corresponds to that part of the solution to equation

(22) $$\begin{array}{c} u\left(t\right)=\left(-\frac{1}{3}-\frac{1}{3}c\right)t+\frac{1}{3}c\frac{1}{t^{2}}+\frac{2}{3}t-\frac{t^{2}}{2}+\frac{t^{4}}{6}, \end{array}$$

for which *c* = 1 and corresponds to a set [0.5; 0.7] × [2.75; 0.4]

(3) CD curve corresponds to that part of the solution to equation

(23) $$\begin{array}{c} u\left(t\right)=\frac{t^{3}}{2}-\frac{1}{3}{ct}^{-2}-\left(1-\frac{1}{3}c\right)t+\frac{1}{2}, \end{array}$$

for which *c* = 3 and corresponds to a set [−2.5; −2] × [−2; −4.9]

(4) DE curve corresponds to that part of the solution to equation

(24) $$\begin{array}{c} u\left(t\right)=\left(-\frac{1}{3}-\frac{1}{3}c\right)t+\frac{1}{3}c\frac{1}{t^{2}}+\frac{2}{3}t-\frac{t^{2}}{2}+\frac{t^{4}}{6}, \end{array}$$

for which *c* = 0 and corresponds to a set [−2.25; 0.9] × [−1.8; −0.9]

(5) EF curve corresponds that part of the solution of the equation

(25) $$\begin{array}{c} u\left(t\right)=\left(-\frac{1}{3}-\frac{1}{3}c\right)t+\frac{1}{3}c\frac{1}{t^{2}}+\frac{2}{3}t-\frac{t^{2}}{2}+\frac{t^{4}}{6}, \end{array}$$

for which *c* = 0 and corresponds to a set [1.5; 0.1] × [2.1; 2.7]

(6) FH curve corresponds to that part of the solution to equation

(26) $$\begin{array}{c} u\left(t\right)=\frac{t^{3}}{2}-\frac{1}{3}{ct}^{-2}-\left(1-\frac{1}{3}c\right)t+\frac{1}{2}, \end{array}$$

for which *c* = 0 and corresponds to a set [−0.7; 1] × [−1.45; 0.6]

(7) HN curve corresponds to that part of the solution to equation

(27) $$\begin{array}{c} u\left(t\right)=\left(-\frac{1}{3}-\frac{1}{3}c\right)t+\frac{1}{3}c\frac{1}{t^{2}}+\frac{2}{3}t-\frac{t^{2}}{2}+\frac{t^{4}}{6}, \end{array}$$

for which *c* = 3 and corresponds to a set [−2.2; −0.55] × [−1.8; 2.6]

(8) NP curve corresponds to that part of the solution to equation

(28) $$\begin{array}{c} u\left(t\right)=\frac{t^{3}}{2}-\frac{1}{3}{ct}^{-2}-\left(1-\frac{1}{3}c\right)t+\frac{1}{2}, \end{array}$$

for which *c* = 2 and corresponds to a set [−0.5; −3.1] × [−2.1; −6.1]

(9) PQ curve corresponds to that part of the solution to equation

(29) $$\begin{array}{c} u\left(t\right)=\left(-\frac{1}{3}-\frac{1}{3}c\right)t+\frac{1}{3}c\frac{1}{t^{2}}+\frac{2}{3}t-\frac{t^{2}}{2}+\frac{t^{4}}{6}, \end{array}$$

for which *c* = 3 and corresponds to a set [1.75; −1.8] × [2.6; 0.1]

(10) QA curve corresponds to that part of the solution to equation

(30) $$\begin{array}{c} u\left(t\right)=\frac{t^{3}}{2}-\frac{1}{3}{ct}^{-2}-\left(1-\frac{1}{3}c\right)t+\frac{1}{2}, \end{array}$$

for which *c* = 5 and corresponds to a set [0.4; 3] × [0.6; 1]

Also, in this case, the mathematical algorithm and the mentioned software were used to construct the geometric shape of the curves to represent the locally over-pressured areas, which are the exact match to the shape of the curve shown in Figure 5.

Figure 6 depicts the curve's geometric shape representing the locally over-pressured area in the left foot's MTP area, taken from the pedogram.

The curve was preliminarily divided into seven parts to describe its shape. Each numbered section was described using the integral curves of solutions to the differential equations given below. Nine parts of the integral curves identically corresponding to the geometric shapes of the curve of the over-pressure area at the point of MTP joints of the left foot were chosen, particularly the following:

1. AB curve corresponds to that part of the solution to equation

(31) $$\begin{array}{c} u\left(t\right)=\left(-\frac{1}{3}-\frac{1}{3}c\right)t+\frac{1}{3}c\frac{1}{t^{2}}+\frac{2}{3}t-\frac{t^{2}}{2}+\frac{t^{4}}{6}, \end{array}$$

for which *c* = 0 and corresponds to a set [2.5; 5.1] × [1.4; 0.1]

(2) BC curve corresponds to that part of the solution to equation

(32) $$\begin{array}{c} u\left(t\right)=\left(-\frac{1}{3}-\frac{1}{3}c\right)t+\frac{1}{3}c\frac{1}{t^{2}}+\frac{2}{3}t-\frac{t^{2}}{2}+\frac{t^{4}}{6}, \end{array}$$

for which *c* = 1 and corresponds to a set [−1; 2.05] × [−0.5; 0]

(3) CD curve corresponds to that part of the solution to equation

(33) $$\begin{array}{c} u\left(t\right)=\frac{t^{3}}{2}-\frac{1}{3}{ct}^{-2}-\left(1-\frac{1}{3}c\right)t+\frac{1}{2}, \end{array}$$

for which *c* = 0 and corresponds to a set [−2.1; −1.6] × [−0.9; 1.1]

(4) DE curve corresponds that part of the solution of the equation

(34) $$\begin{array}{c} u\left(t\right)=\left(-\frac{1}{3}-\frac{1}{3}c\right)t+\frac{1}{3}c\frac{1}{t^{2}}+\frac{2}{3}t-\frac{t^{2}}{2}+\frac{t^{4}}{6}, \end{array}$$

for which *c* = 2 and corresponds to a set [−2.5; 5.9] × [−2; 2.4]

(5) EF curve corresponds to that part of the solution to equation

(35) $$\begin{array}{c} u\left(t\right)=\frac{t^{3}}{2}-\frac{1}{3}{ct}^{-2}-\left(1-\frac{1}{3}c\right)t+\frac{1}{2}, \end{array}$$

for which *c* = 5 and corresponds to a set [−0.8; −3.5] × [−0.7; −5.2]

(6) FH curve corresponds to that part of the solution to equation

(36) $$\begin{array}{c} u\left(t\right)=\left(-\frac{1}{3}-\frac{1}{3}c\right)t+\frac{1}{3}c\frac{1}{t^{2}}+\frac{2}{3}t-\frac{t^{2}}{2}+\frac{t^{4}}{6}, \end{array}$$

for which *c* = 5 and corresponds to a set [−0.6; 3.2] × [−0.95; 0.8]

(7) HN curve corresponds to that part of the solution to equation

(37) $$\begin{array}{c} u\left(t\right)=\frac{t^{3}}{2}-\frac{1}{3}{ct}^{-2}-\left(1-\frac{1}{3}c\right)t+\frac{1}{2}, \end{array}$$

for which *c* = 5 and corresponds to a set [−1.9; −1.1] × [−0.7; 0.15]

(8) HP curve corresponds to that part of the solution of the equation

(38) $$\begin{array}{c} u\left(t\right)=\left(-\frac{1}{3}-\frac{1}{3}c\right)t+\frac{1}{3}c\frac{1}{t^{2}}+\frac{2}{3}t-\frac{t^{2}}{2}+\frac{t^{4}}{6}, \end{array}$$

for which *c* = 0 and corresponds to a set [−0.5; −0.45] × [0.6; 0]

(9) PA curve corresponds to that part of the solution to equation

(39) $$\begin{array}{c} u\left(t\right)=\frac{t^{3}}{2}-\frac{1}{3}{ct}^{-2}-\left(1-\frac{1}{3}c\right)t+\frac{1}{2}, \end{array}$$

for which *c* = 0 and corresponds to a set [1.8; 2] × [1.55; 1.9]

The mathematical algorithm and the software developed within this research for construction of the geometric shape of the curves were used to represent the locally over-pressured areas. The exact image is shown in Figure 6.

Figure 7 geometrically shows the curve of the locally over-pressured areas in the heel area of the left foot, taken from the pedogram.

The curve was preliminarily divided into seven parts to describe its shape. Each numbered section was described using the integral curves of solutions to differential equations given below. The seven parts of the integral curves identical to the geometric shapes of the curve of the over-pressure region in the heel area of the left foot were chosen, particularly the following:

1. AB curve corresponds to that part of the solution to equation

(40) $$\begin{array}{c} u\left(t\right)=\frac{t^{3}}{2}-\frac{1}{3}{ct}^{-2}-\left(1-\frac{1}{3}c\right)t+\frac{1}{2}, \end{array}$$

for which *c* = 2 and corresponds to a set [−2.4; −8.5] × [−1.1; −2.4]

(2) BC curve corresponds to that part of the solution to equation

(41) $$\begin{array}{c} u\left(t\right)=\left(-\frac{1}{3}-\frac{1}{3}c\right)t+\frac{1}{3}c\frac{1}{t^{2}}+\frac{2}{3}t-\frac{t^{2}}{2}+\frac{t^{4}}{6}, \end{array}$$

for which *c* = 0 and corresponds to a set [−1.7; −0.8] × [−2.5; 2]

(3) CD curve corresponds to that part of the solution to equation

(42) $$\begin{array}{c} u\left(t\right)=\frac{t^{3}}{2}-\frac{1}{3}{ct}^{-2}-\left(1-\frac{1}{3}c\right)t+\frac{1}{2}, \end{array}$$

for which *c* = 0 and corresponds to a set [−1.2; −2.5] × [−1.3; 0.8]

(4) DE curve corresponds to that part of the solution to equation

(43) $$\begin{array}{c} u\left(t\right)=\frac{t^{3}}{2}-\frac{1}{3}{ct}^{-2}-\left(1-\frac{1}{3}c\right)t+\frac{1}{2}, \end{array}$$

for which *c* = 5 and corresponds to a set [−2.25; −3.8] × [1; 0.2]

(5) EF curve corresponds to that part of the solution to equation

(44) $$\begin{array}{c} u\left(t\right)=\left(-\frac{1}{3}-\frac{1}{3}c\right)t+\frac{1}{3}c\frac{1}{t^{2}}+\frac{2}{3}t-\frac{t^{2}}{2}+\frac{t^{4}}{6}, \end{array}$$

for which *c* = 0 and corresponds to a set [2.05; 1.9] × [1; 0.05]

(6) FH curve corresponds to that part of the solution to equation

(45) $$\begin{array}{c} u\left(t\right)=\left(-\frac{1}{3}-\frac{1}{3}c\right)t+\frac{1}{3}c\frac{1}{t^{2}}+\frac{2}{3}t-\frac{t^{2}}{2}+\frac{t^{4}}{6}, \end{array}$$

for which *c* = 1 and corresponds to a set [−0.5; 0.1] × [−0.8; 2.5]

(7) HA curve corresponds to that part of the solution to equation

(46) $$\begin{array}{c} u\left(t\right)=\left(-\frac{1}{3}-\frac{1}{3}c\right)t+\frac{1}{3}c\frac{1}{t^{2}}+\frac{2}{3}t-\frac{t^{2}}{2}+\frac{t^{4}}{6}, \end{array}$$

for which *c* = 3 and corresponds to a set [−0.55; 4] × [−0.95; 0.85]

Based on the mathematical algorithm and the software, the geometric shape of the curves was constructed to show the locally over-pressured areas. The exact image is shown in Figure 7.

Through the integral curves of the solutions to the Dirichlet singular boundary problem, it is possible to describe the geometric shape of a curve of any complexity with high precision that will be registered as the over-pressure area on the pedograms of the patients with diabetic foot.

Thus, based on the use of the pedograph and the mathematical research methods, the study describes the complex geometric figures of the over-pressure areas presented on the pedogram.

## 4. Discussion

The process of design and manufacture of individual orthopedic insoles is quite complicated and sequential. In the paper, the pedogram of the patient with diabetic foot is presented, on which the over-pressure areas are marked with the curved lines. Based on the analysis of the pedogram, it was established that the pressure on the over-pressure areas ranges from 220 to 400 kPa. The peak pressure on the right foot is 390 kPa, and on the left foot, it is 355 kPa, which is unacceptable for patients with diabetic foot. Those areas are considered as the areas of risk, where the diabetic ulcers develop over time. As shown in Figure 3, both feet have the over-pressure areas, both in the heel part and in the metatarsophalangeal (MTP) joints.

The curves with complex geometric shape of the locally over-pressured areas presented on the pedogram are described through the integral curves of the solutions to the Dirichlet singular boundary problem. The mathematical algorithm describing the curves with complex geometric shapes of the over-pressure areas on the pedogram was designed for all over-pressure areas of the feet, which is shown in Figures 4–7. Based on this mathematical algorithm, the complete software packages were developed, on the basis of which individual orthopedic insoles were produced on the CNC milling machine Ped-Cad Foot Technology (Oberkochen, Germany), taking into account the local pressures on the plantar side of the foot, which is shown in Figure 8.

The complex geometrical shapes were produced on a CNC-milling machine using the soft material—EVA polymer—with the hardness of 20 Shore A (the white material in Figure 8). The main frame of the insole was made with the EVA polymer, the hardness of which was up to 40 Shore A (the green material in Figure 8). Further, the milled parts of the locally over-pressured areas were preliminarily inserted (the white material in Figure 8) into the main frame of the insole (the green material in Figure 8) separately. Finally, the complete insole was manufactured on the CNC-milling machine simultaneously taking into account the locally over-pressured areas as presented in Figure 8.

For preparation of CMI (custom-made insole), a 3D model of the foot was developed [21]. The materials of different degrees of hardness and thickness and their combinations were examined by the method of FEA (finite element analysis) to reduce the peak contact pressure of the diabetic foot with neuropathy. Application of soft materials (EVA) tends to effectively reduce the peak contact pressure compared to the harder material of thermopolyurethane (TPU). CMI, produced either from the soft material alone or from a combination of the soft and hard materials, reduce the peak contact pressure of the plantar side of the foot.

Application of the mathematical method of research makes it possible to describe the similarities; the reduction of the peak contact pressure was observed in the case of application of different shock-absorbing materials compared to the flat insoles [22]. Reduction of the peak pressure is considered in [23], where the optimal range of constructive parameters of the insoles is investigated by the method of FEA. It is established that the shape of the insoles significantly affects the peak pressure and the distribution of pressure on the plantar sides of the feet. The results of the study show that the insole made according to the individual order reduces the peak pressure by 40% more than the insole with a flat surface. In addition, the insole made according to the individual order evenly distributes the pressure over the plantar sides of the foot compared to the flat insole.

It should be noted that, in contrast to the existing studies, the present work uses a mathematical research method that allows describing the shape of the congested areas of the plantar side of the diabetic foot with great accuracy. Individual orthopedic insoles manufactured taking into account the over-pressure areas of the foot effectively reduce pressure in the risk areas, increase the contact area, and redistribute pressure to other areas of the foot.

Individual orthopedic insoles manufactured using this method will protect the diabetic foot from mechanical injuries and development of ulcers. Practical application of these methods and their implementation into production will facilitate the effective treatment of patients with diabetic foot.

## 5. Conclusions

Based on the pedographic study of the patients with diabetic foot, the locally over-pressured areas of the plantar side of the foot were identified and shaped by curves. The curves of complex geometric shapes of the over-pressure areas were described on each patient's pedograms by the integral curves of the solutions to Dirichlet singular boundary differential equations with great accuracy. Based on the mathematical algorithm, the software package was developed to describe the above curves. Individual orthopedic insoles were manufactured on a CNC-controlled milling machine with combined materials considering the locally over-pressured areas.

The soft material used for production of individual orthopedic insoles for the over-pressure areas helps the reduction of the pressure on the plantar side of the foot and increases the contact area. A relatively hard material used as the main frame imparts the stability to the insole shape and increases its wear life. Application of combined materials for designing and manufacturing of the individual orthopedic insoles with account of locally over-pressured areas on the plantar side of the foot is particularly relevant for the patients with diabetic foot.

It is necessary to continue the research in the direction of selection of polymeric materials of different degrees of hardness in order to further improve the comfort of the insole.

## Figures and Tables

**Figure 1:** The curves of the solutions.

**Figure 2:** The curves of the solutions.

**Figure 3:** The pedogram of a patient with diabetic foot.

**Figure 4:** The curve's shape of the locally over-pressured area in the right foot's MTP.

**Figure 5:** The curve's shape of the locally over-pressured area in the right foot's heel area.

**Figure 6:** The curve's shape of the locally over-pressured area in the left foot's MTP area.

**Figure 7:** The curve's shape of the locally over-pressured area in the left foot's heel area.

**Figure 8:** The individual orthopedic insoles, taking into account the locally over-pressured areas on the plantar side of the foot.

## Data Availability

The data during the current study are available from the corresponding authors on request.

## References

[1] Hess C. T. (2020). Diabetic foot ulcer assessment and management: use of classification systems for healing progress. *Advances in Skin & Wound Care*.

[2] Senneville E., Joulie D., Blondiaux N., Robineau O. (2020). Surgical techniques for bone biopsy in diabetic foot infection, and association between results and treatment duration. *Journal of Bone and Joint Infection*.

[3] Bus S. A., Armstrong D. G., van Deursen R. W. (2016). IWGDF guidance on footwear and offloading interventions to prevent and heal foot ulcers in patients with diabetes. *Diabetes/Metabolism Research and Reviews*.

[4] Reiber G. E., Smith D. G., Wallace C. (2002). Effect of therapeutic footwear on foot reulceration in patients with diabetes: a randomized controlled trial. *Journal of the American Medical Association*.

[5] Paton J. S., Stenhouse E. A., Bruce G., Zahra D., Jones R. B. (2012). A comparison of customised and prefabricated insoles to reduce risk factors for neuropathic diabetic foot ulceration: a participant-blinded randomised controlled trial. *Journal of Foot and Ankle Research*.

[6] van Netten J. J., Lazzarini P. A., Armstrong D. G. (2018). Diabetic Foot Australia guideline on footwear for people with diabetes. *Journal of Foot and Ankle Research*.

[7] Martinez-Santos A., Preece S., Nester C. J. (2019). Evaluation of orthotic insoles for people with diabetes who are at-risk of first ulceration. *Journal of Foot and Ankle Research*.

[8] Gao Y., Wang C., Chen D. (2021). Effects of novel diabetic therapeutic footwear on preventing ulcer recurrence in patients with a history of diabetic foot ulceration: study protocol for an open-label, randomized, controlled trial. *Trials*.

[9] Ahmed S., Barwick A., Butterworth P., Nancarrow S. (2020). Footwear and insole design features that reduce neuropathic plantar forefoot ulcer risk in people with diabetes: a systematic literature review. *Journal of Foot and Ankle Research*.

[10] Skidan V., Nadopta T., Mytelska O., Yefimchuk H., Stetsiuk I., Yanovets A. (2019). Method of sketch profiling with spline curves for footwear design. *Leather and Footwear Journal*.

[11] Driscu M. (2010). A method to approximate a spatial surface using a Bézier bi-cubic surface. *Revista de Pielarie Incaltaminte*.

[12] Zamarashkin K., Zamarashkin N. (2009). Design of shoe lasts with variable forepart. *Footwear Science*.

[13] Zamarashkin K., Zamarashkin N. (2009). Reference coordinate system in design of shoe lasts. *Footwear Science*.

[14] Shalamberidze M., Sokhadze Z. (2018). Constructing a shape of orthopedic boot-tree print by means of the solution to differential equation with deviating argument. *ISJ Theoretical & Applied Science*.

[15] Shalamberidze M., Sokhadze Z., Tatvidze M. (2018). Construction of the transverse-vertical shapes of the orthopedic boot tree by means of the solution to singular Dirichlet boundary value problem. *Bulletin of the Georgian National Academy of Sciences*.

[16] Shalamberidze M., Sokhadze Z., Tatvidze M. (2019). Construction of the orthopedic boot-tree print and main longitudinal-vertical section by means of the solution of differential equations. *Bulletin of the Georgian National Academy of Sciences*.

[17] Gerrard J. M., Bonanno D. R., Whittaker G. A., Landorf K. B. (2020). Effect of different orthotic materials on plantar pressures: a systematic review. *Journal of Foot and Ankle Research*.

[18] Rachůnková I., Spielauer A., Staněk S., Weinmüller E. B. (2013). The structure of a set of positive solutions to Dirichlet BVPs with time and space singularities. *Georgian Mathematical Journal*.

[19] Shalamberidze M., Sokhadze Z., Tatvidze M. (2020). Orthopedic boot-tree 3D design by means of the integral curves of solutions of differential equations. *Complexity*.

[20] Shalamberidze M., Sokhadze Z., Tatvidze M. (2019). Construction of the main transverse-vertical cross-sections for orthopedic shoe trees and 3D design of the shoe tree frame. *Bulletin of the Georgian National Academy of Sciences*.

[21] Nouman M., Dissaneewate T., Chong D. Y. R., Chatpun S. (2021). Effects of custom-made insole materials on frictional stress and contact pressure in diabetic foot with neuropathy: results from a finite element analysis. *Applied Sciences*.

[22] Goske S., Erdemir A., Petre M., Budhabhatti S., Cavanagh P. R. (2006). Reduction of plantar heel pressures: insole design using finite element analysis. *Journal of Biomechanics*.

[23] Sarikhani A., Motalebizadeh A., Asiaei S., Kamali Doost Azad B. (2016). Studying maximum plantar stress per insole design using foot CT-scan images of hyperelastic soft tissues. *Applied Bionics and Biomechanics*.

